# Estimation of Copper and Cadmium Bioavailability in Contaminated Soil Remediated by Different Plants and Micron Hydroxyapatite

**DOI:** 10.1155/2022/3565550

**Published:** 2022-06-06

**Authors:** Lei Xu, Xiangyu Xing, Jianbiao Peng, Mingfei Ji

**Affiliations:** ^1^Key Laboratory of Natural Disaster and Remote Sensing of Henan Province, Nanyang Normal University, Nanyang 473061, China; ^2^Henan Key Laboratory of Ecological Security for Water Source Region of Mid-line of South-to-North Diversion Project, Nanyang Normal University, Nanyang 473061, China; ^3^College of Non-Major Foreign Language Teaching, Nanyang Normal University, Nanyang 473061, China; ^4^School of Environment, Henan Normal University, Xinxiang 453007, China

## Abstract

A three-year in situ remediation experiment was carried out to understand the effect of combined phytoremediation with chemical materials on the bioavailability of heavy metals in soil. Indigenous weed (Setaria pumila), energy plant (Pennisetum sp.), cadmium (Cd)-hyperaccumulator (Sedum plumbizincicola), and copper (Cu)-tolerant plant (Elsholtzia splendens) were used as the phytoremediation plants aided by micron hydroxyapatite (1% wt). The bioavailability of Cu and Cd in soil was evaluated during the three years. The results showed that the four plants combined with micron hydroxyapatite significantly increased soil pH and soil organic carbon (SOC), and decreased Cu and Cd fractions extracted by CaCl_2_ and diffusive gradients in thin films (DGT) than the untreated soils, respectively. Because of the large biomass, the accumulation of Cu and Cd is the largest in Pennisetum sp. followed by Elsholtzia splendens, Sedum plumbizincicola, and Setaria pumila. The bioavailability of Cu and Cd is significantly negatively correlated with pH, soil organic carbon, available phosphorus, and available potassium. Moreover, the correlation is mainly related to the addition of micron hydroxyapatite. The accumulation of Cu and Cd is the combined action of the soil bioavailability of Cu, Cd, and biomass. Our results suggest that Pennisetum sp. can act as an appropriate remediation plant for phytoremediation aided by amendments.

## 1. Introduction

During the past few decades, elevating Cu and Cd concentrations in Chinese arable soils due to industrial and agricultural activities represents a serious threat to humans [1]. Thus, remediation of metal-contaminated agricultural soils has been widely carried out in China [2]. Phytoextraction as an environmentally friendly and cost-effective technique has been widely used to remediate the heavy metal- contaminated soil [3]. However, excessive soil pollutants with adverse physical and chemical properties in seriously contaminated soil may lead to cause poisoning symptoms of plants and inhibit its growth, so as to limit the remediation process [4]. Therefore, the application of inorganic and/or organic chemical materials to assist phytoremediation in heavy metal severely contaminated soil is widely advocated [5] because this method can improve the physicochemical and biological properties of soil and thus promoting plant growth [6]. The objective of aiding phytoremediation is not only to remove heavy metals from soil but also to decrease the bioavailability of heavy metals in soil, so as to decrease their potential environmental risks [5]. Additionally, the bioavailability of heavy metals during the phytoremediation is primarily associated with the phytotoxicity of trace metals in soil [7]. Therefore, it is of great significance to accurately evaluate the bioavailability of heavy metals in soil during phytoremediation aided by soil amendments.

It has been reported that some hyperaccumulator plants, agricultural grasses, and energy plants with high productivity can be used for phytoremediation because they can absorb heavy metals from soil [8]. However, high metal availability, low soil pH, organic matter (OM) and nutrients, and poor soil structure in contaminated soils could also prevent plant establishment and growth [9]. Therefore, appropriate soil amendments such as limestone, apatite, and zeolite have been applied to enhance plant biomass production [10]. For example, Gray et al. found that red fescue (Festuca rubra) could be only established in heavy metal-contaminated soil with the applications of lime and red mud [11]. On the other hand, the process of plant uptake of heavy metals in soil may be affected by the addition of chemical materials, thus reducing the efficiency of phytoremediation [12]. In phytoremediation, a great deal of studies suggested that soil amendments play more important roles in decreasing the bioavailability of heavy metals compared with plants [13, 14]. To date, however, it is not clear that the bioavailability of heavy metals to different plant species during phytoremediation aided by the same amendment. It has been reported that micron hydroxyapatite has strong fixation ability for heavy metals [15] and is widely used to remediate heavy metal-contaminated soil. Although this stabilizing remediation method cannot reduce the total amount of heavy metals, it can combine with heavy metals or transform them from active state to inactive state. In addition, some studies showed that hydroxyapatite had the characteristics of low leaching rate and slow phosphorus release compared with conventional water-soluble phosphate fertilizer, which made it a potential phosphate fertilizer in China [16]. Therefore, the application of hydroxyapatite in the red soil contaminated by heavy metals in China can not only reduce the activity of heavy metals but also promote the growth of crops.

Many methods have been used to evaluate the bioavailability of Cu and Cd, mainly including chemical extraction and some other methods such as the diffusive gradients in thin films (DGT). The dissolved part of heavy metals in soil is considered to have the highest bioavailability [17], 0.01 mol L^−1^ CaCl_2_ often be used to extract the dissolved part metal fraction in soil [18]. As a kinetically based technique, DGT can reflect the soil metal desorption process when metals in the soil solution are depleted at the interface between the roots and the soil [19]. Meanwhile, the bioavailability of heavy metals in soil always substantially affected by soil physicochemical properties, and this effect is not only reflected in the mobility of heavy metals in soil but also reflected in the impact on plant growth and soil structure, thus affecting the efficiency of phytoremediation [20]. Among many physicochemical properties, the soil pH, soil organic matter (SOM), nutritional status, and texture play important roles in plant growth, thus affecting the remediation efficiency [21–24]. The phytoremediation aided by remediation materials will affect the bioavailability of heavy metals in the soil and the soil physicochemical properties, making the relationship between remediation efficiency and soil factors more complex. Thus, it is necessary to find a method to describe quantitatively the contribution of individual variables to Cu and Cd bioavailability and remediation efficiency in the complex ecosystems of soils.

In the present study, a three-year field experiment was conducted by adding micron hydroxyapatite into the co-contaminated soil (Cu and Cd) and planting four plant species. The aims were (i) to assess the bioavailability of Cu and Cd to different plant species using two extraction methods (0.01 mol L^−1^ CaCl_2_ and DGT), (ii) to quantify the contribution rates of different soil properties to Cu and Cd bioavailability, and remediation efficiency, and (iii) finally to provide some suggestions for the practical use of heavy metal accumulators aided by amendment in decontaminating metal-contaminated agricultural soils in China.

## 2. Materials and Methods

### 2.1. Study Site

The field experiment was conducted in Guixi City, Jiangxi Province, China (116°55′ E, 28°12′ N). Owing to farmers using wastewater containing heavy metals discharged by a copper smelter for irrigation and the atmospheric metal depositions, and waste residue accumulation, more than 130 hm^2^ of surrounding farmland has suffered heavy metal pollution (mainly Cu and Cd). The soil texture is sandy loam, and the main soil properties are shown in Table 1.

### 2.2. Reagent and Plants

Micron hydroxyapatite (purity >96.0%, pH 7.71) was purchased from Emperor Nano Material Co. Ltd (Nanjing, China), and the major properties have been listed in our previous research [25]. The remediation plants used in this study were Elsholtzia splendens, Sedum plumbizincicola, Pennisetum sp., and an indigenous weed (Setaria lutescens). These plant species were selected because Sedum plumbizincicola is a Cd-hyperaccumulator [26]; Elsholtzia splendens is a Cu-tolerant species [27], Pennisetum sp. is high biomass species [28], and Setaria lutescens is a native weed. Moreover, Sedum plumbizincicola and Pennisetum sp. are perennial species, while Elsholtzia splendens and Setaria lutescens are annual species.

### 2.3. Plot Design

The experiment included five treatments: control soil without micron hydroxyapatite and plant (CK), 1% micron hydroxyapatite combined with native Setaria lutescens and without manual planting (MW), 1% micron hydroxyapatite and Elsholtzia splendens (ME) with planting density of 20 cm × 20 cm, 1% micron hydroxyapatite and Sedum plumbizincicola (MS) with planting density of 20 cm × 20 cm, and micron hydroxyapatite and Pennisetum sp. (MP) with planting density of 50 cm × 50 cm. Each plot was 500 cm (length) × 400 cm (width) and received one application of 1% micron hydroxyapatite (based on the 0–17 cm soil weight) and 834 kg ha^−1^ fertilizer (the content of N-15%, P_2_O_5_-15%, K_2_O-15%) on December 23, 2012, and the micron hydroxyapatite and fertilizer fully mixed into the soil by plowing. The plants were planted on April 26 each year (2013, 2014, and 2015), and the micron hydroxyapatite was applied once in 2012, but fertilizer was added into soil each year for the next three years.

### 2.4. Sample Collection

All the plants' shoots were harvested in December 15 each year except Sedum plumbizincicola, which was harvested in July 15 each year. Five top-soil samples (about 1 kilogram) near the plant rhizosphere were collected from the 0–17 cm depth each year. Then, the five samples were mixed and formed a composite sample for the physicochemical analysis.

### 2.5. Soil Physicochemical Analysis

Soil pH was measured with a glass electrode in water: soil ratio of 2.5 : 1(PHS-2CW-CN, Bante, Shanghai, China). Soil organic carbon (SOC) and total nitrogen (TN) were determined according to Walkley–Black [29]. Soil available phosphate (P) and nitrogen (N) were measured in accordance with Holliday [30]. The soil available potassium (K) was measured in accordance with Olsen [31, 32]. The ammonium acetate method was used to measure the soil cation exchange capacity (CEC) [33].

### 2.6. Heavy Metal Analysis

#### 2.6.1. Heavy Metals Concentrated by DGT

The technique of diffusive gradients in thin films (DGT) continuously removes metal to the resin sink after it diffuses through a hydrogel [34]. It mimics the processes of metal uptake by plants that occur in the rhizosphere including soil solution metal resupply from the solid phase at the time scale of plant metal uptake [35]. The DGT technique has been used for several decades to study metal bioavailability, and good correlations have been obtained between metal measured by DGT and metal in metal-tolerant plants or crops. Standard piston DGT devices (DGT Research, Lancaster, UK) were prepared with a diffusion layer overlying a Chelex (Bio-Rad, Hercules, CA) resin layer. The diffusion layer was composed of a 0.8-mm-thick polyacrylamide gel with agarose derivative cross-linker and a 0.13-mm-thick 0.45-mm cellulose nitrate filter. For DGT measurements, 30-g air-dried soil was weighed into a small plastic beaker and maintained approximately 70% of the maximum water-holding capacity for 48 h at 25°C in order to ensure sufficient moisture for the assay. Then, the soil moisture content was adjusted to 100% field capacity and the soil was mixed thoroughly using a plastic spatula until a smooth paste was formed. The soil paste was left to equilibrate for 1 day at room temperature (18–20°C) before DGT deployment. The DGT devices were placed carefully on the soil paste with slight pressure to ensure complete contact between the filter membrane of each device and the soil. The acid soils (DBS and HLD) were deployed for 16 h at 19 ± 1°C, and on the alkaline soil (where the metals had low availabilities), DGT devices were deployed for 24 h. On retrieval, the surfaces of the DGT devices were jet-washed with deionized water to remove soil particles and then disassembled. 1 mL of HNO_3_ (1 M) was added in a closed microvial to elute the metal from the resin gel. After retrieval of the DGT device, the paste soil was stirred and centrifuged at 3000 rpm for 30 min to collect the soil solution. The supernatant was syringe-filtered using 0.45-mm disposable polysulfone filter assemblies and acidified using 10 mL of 5 M HNO_3_ in 1 mL. Eluted metals and metals in the soil solution were measured by atomic absorption spectrophotometry (AAS, SpectrAA-220, Varian Medical Systems, Palo Alto, CA, USA).

The mass of metal accumulated (*M* in mg) in the resin gel layer of DGT was obtained by the following formula:

(1) $$\begin{array}{c} M=\frac{C_{E}\left(V_{{\text{HNO}}_{3}}\;+\;V_{\text{gel}}\right)}{f_{e}}, \end{array}$$

where *C*_*E*_ is the concentration of metal in the 1 M HNO_3_ elution solution (*μ*g L^−1^); VHNO3 is the volume of HNO_3_ added to the resin gel (1 mL); *V*_gel_ is the volume of the resin gel, typically 0.15 mL; and *f*_*e*_ is the elution factor for each metal, typically 0.8.

The flux of metal measured by DGT (*F*, in *μ*g cm^−2^ s^−1^) and the concentration of metal at the interface of the DGT device and the soil (*C*_DGT_ , in *μ*g L^−1^) were calculated as follows:

(2) $$\begin{array}{c} F=\frac{M}{\left(tA\right)}, \end{array}$$

(3) $$\begin{array}{c} C_{\text{DGT}}=\frac{F\Delta g\;}{D}, \end{array}$$

where *t* is the DGT deployment time (in sec); *A* is the contact area between soil and diffusive layer, typically 2.54 cm^2^; Δ*g* is the diffusive thickness (0.094 cm); and *D* is the diffusion coefficient of the metal in the gel (cm^2^ s^−1^).

#### 2.6.2. Heavy Metals Extracted by Chemical Agents

5 g of soil sample was weighed and added into 50-mL centrifuge tube, and then, 25 mL of 0.01 mol L^−1^ CaCl_2_ solution was added into the tube and shake at 25°C for 2 h, then centrifuged at 3500 rpm for 5 min; subsequently, the supernatant was filtered by 0.45-*μ*m micron microporous filter membrane. Atomic absorption spectrophotometry (AAS, SpectrAA-220, Varian Medical Systems, Palo Alto, CA, USA) was used to determine the Cu and Cd concentrations in the supernatant.

#### 2.6.3. Determination of Heavy Metals in Soil and Plant Sample

Total soil Cu and Cd in soil and plant were measured by atomic absorption spectrophotometry (AAS, SpectrAA-220, Varian Medical Systems, Palo Alto, CA, USA). Standard soil samples (GBW07405, National Research Center for Certified Reference Materials, Beijing, China; GBW07401, Institute of Geophysical and Geochemical Exploration, Langfang, Hebei Province, China) were used to verify data reliability.

### 2.7. Statistical Analysis

All the data were presented as mean standard error and were estimated using one-way ANOVA at a significance level of 0.05 using SPSS 20.0 (IBM SPSS, Somers, NY, USA) when necessary and the Pearson's correlation also be analyzed by SPSS 20.0. All the graphics in this article were made with SigmaPlot 12.5.

## 3. Results and Discussion

### 3.1. Surface Soil Properties

The soil pH was significantly increased from 4.24 to 5.17 after the applying of micron hydroxyapatite in the first year (Table 2). This might be due to the high pH (8.40) of micron hydroxyapatite, and the result was consistent with Cui et al., who found that the soil pH could be improved because of the addition of micron hydroxyapatite [36]. However, just as the CK whose pH decreased from 4.24 to 4.20 during the three years (Table 2), the effect of micron hydroxyapatite on the improving soil pH also decreased year by year (Table 2). This might be related to the fact that our experimental area was located in a typical acid rain area in southern China; with a large number of H^+^ entering the soil, the soil pH decreased slightly over time. Although the plants might have secreted some weak organic acid ions, amino acids, vitamins, and inorganic ions (HCO3^−^, OH^−^, and H^+^) by the roots, which could change the soil pH [37], there was no significant difference in soil pH among different plant treatments, implying that the addition of micron hydroxyapatite played a decisive role in the soil pH during the remediation of this contaminated soil. The SOC could be increased significantly by the combined effect of micron hydroxyapatite and Elsholtzia splendens, Sedum plumbizincicola, and Pennisetum sp. in 2014 and 2015 (Table 2). However, only adding micron hydroxyapatite without artificial planting plants (MW) did not significantly improve SOC applying hydroxyapatite alone (MW). This was mainly because the growth of plants increased the input of litter and the number of plant fine roots, which changed the structure of soil aggregates. Soil aggregates had physical protection effect on SOC and reduced the mineralization and decomposition of organic carbon, resulting in the increase of SOC [38]. Because of the addition of micron hydroxyapatite, the total phosphorus and available phosphorus were significantly increased in all the treatments. The soil phosphorus content in southern China is low, which usually made it a limiting factor for plant growth [39], and the addition of micron hydroxyapatite had a significant effect on alleviating the phosphorus shortage in this contaminated soil. Additionally, the addition of micron hydroxyapatite could not significantly increase the content of total N, total K, and available N; however, there were significant change observed among different treatments in terms of available K.

### 3.2. Total and Available Metals and Metals' Supply

The Cu and Cd concentrations in the soils without phytoextraction (CK) and the soils after different phytoextractions are shown in Figure 1. Both soil Cu and Cd did not decrease significantly after remediation in the first 2 years; however, the total Cu and Cd in soil were significantly reduced by all the phytoremediation except Setaria lutescens after the third year of remediation. This might be due to the decrease of biological activity of Cu and Cu in the soil after the addition of micron hydroxyapatite, which reduced the absorption of Cu and Cd by the plants [40]. Therefore, the total Cu and Cd in the soil were not significantly reduced in the remediation in the first 2 years. With the progress of remediation, the stabilization effect of the hydroxyapatite on Cu and Cd in the soil decreased, the biological activity of Cu and Cd in the soil increased, and the absorption of Cu and Cd by plants increased, which significantly improved the remediation effect, so that the concentration of total Cu and Cd in the remediation soil was significantly lower than that in CK [41]. The largest decrease of Cu and Cd occurred in Elsholtzia splendens (ME), Sedum plumbizincicola (MS), and Pennisetum sp. (MP), respectively. And after phytoextraction, the decreases in Cu and Cd were from 10.0 to 52.0 and 0.017 to 0.056 mg kg^−1^, respectively.

It is known that the toxicity of heavy metals in soil mainly depends on its bioavailability, and CaCl_2_-extractable heavy metals have been used to evaluate the bioavailability of heavy metals in soil [42]. The CK had the highest CaCl_2_ extract ability among all the treatments (Cu 81.6 mg·kg^−1^ and Cd 0.125 mg·kg^−1^ in 2013). The CaCl_2_ extract ability had been significantly reduced because of the addition of micron hydroxyapatite; the lowest CaCl_2_-extractable Cu was found in Sedum plumbizincicola plots (22.8 mg·kg^−1^ in 2013; 26.0 mg·kg^−1^ in 2014; and 43.5 mg·kg^−1^ in 2015) and the lowest CaCl_2_-extractable Cd was found in Sedum plumbizincicola plots in 2013 and 2014 (0.066 mg·kg^−1^ and 0.068 mg·kg^−1^) but was found in Pennisetum sp. plots in 2015 (0.089 mg·kg^−1^) (Figures 2(a) and 2(b)). The results implied that the bioavailability of Cu and Cd could be significantly reduced by the application of micron hydroxyapatite. Meanwhile, different plants had different effects on the bioavailability of Cu and Cd in soil during the combined remediation, which could not be ignored.

The results of DGT analysis showed that the addition of micron hydroxyapatite could significantly reduce the DGT concentration of Cu and Cd in soil (Figures 2(c) and 2(d)). The reduction range for Cu and Cd in different years was 46.4%–74.8% and 50.3%–63.3%, respectively. Treatment with the greatest decreased percent for Cu and Cd was Elsholtzia splendens (ME: 74.8%, 2013) and Sedum plumbizincicola (MS: 63.3%, 2013), respectively. However, although different plants had different effects on the DGT concentration of Cu and Cd, there was no significant difference among the different plant treatments. It is noteworthy that the concentrations of available Cu and Cd in soil increased gradually with the passage of time. Due to the changes of soil physical and chemical properties, the remediation effect of the amendment will gradually decrease over time, and the heavy metals originally fixed by the amendment or inactive heavy metals in the soil would be released again. This might be due to the influence of acid deposition in this area, which reduced the soil pH value and weakened the adsorption capacity of soil minerals to heavy metals [43]. Other types of research also found that the stabilizing effect of amendment on heavy metals decreased gradually with the passage of time through the simulation test of 6 years [44, 45].

Through the analysis of Cu and Cd extracted by CaCl_2_ and DGT in soil, it was found that the bioavailability of Cu and Cd in soil is significantly reduced after the soil is remediated by micron hydroxyapatite. This phenomenon may be related to four mechanisms: firstly, phosphate induces heavy metal adsorption. On variable charge soil, because it is rich in iron oxide, alumina, and kaolinite, it can specifically adsorb phosphate, resulting in the increase of negative charge on the soil surface and/or the increase of solution pH, so as to induce the increase of heavy metal adsorption and reduce the bioavailability of soil heavy metals [15, 46, 47]. Secondly, in most soils with high content of heavy metals, the addition of micron hydroxyapatite can form heavy metal phosphate precipitation or minerals with heavy metals in the soil, so as to reduce the bioavailability of heavy metals in the soil [48, 49]. Thirdly, the micron hydroxyapatite added to the soil directly adsorbs heavy metals. Because the solubility of micron hydroxyapatite is small and the specific surface area of micron hydroxyapatite is large, after adding to the soil, some heavy metal ions will be adsorbed on the surface of micron hydroxyapatite, thus reducing the bioavailability [50, 51]. Additionally, four plant species may also stabilize Cu and Cd by their absorption and accumulation in roots [52].

However, it is found that planting different plants in the soil with remediated by micron hydroxyapatite has no significant difference in the bioavailability of soil Cu and Cd, which is different from other research results. For example, Li et al. found that continuous planting of Sedum plumbizincicola in Cd polluted soil can reduce the CaCl_2_-extractable Cd and DGT Cd by 60% and 82%, respectively [53]. This may be because in our study, micron hydroxyapatite was added for remediation to reduce the toxicity of Cu and Cd in soil, and then, different plants were planted. The addition of hydroxyapatite reduces the bioavailability of Cu and Cd in soil, thus reducing the ability of plants to absorb and accumulate for Cu and Cd. This also led to no significant difference in the effects of different plants on the bioavailability of Cu and Cd in soil. The phytoremediation using different plants aided by micron hydroxyapatite, which seems to reduce the phytoremediation efficiency, but it is of great significance to the ecological restoration of heavy metal-contaminated areas.

### 3.3. Plant Biomass and Metal Concentrations in Plants

The native grass Setaria lutescens and three phytoextractors could grow normally after the application of micron hydroxyapatite; however, there was no plant growth in CK treatment without micron hydroxyapatite. There were significant differences in the biomass of the four plants, the largest was found in Pennisetum sp., and biomass of Elsholtzia splendens was smaller than that of Pennisetum sp. but significantly higher than that of Setaria lutescens and Sedum plumbizincicola (Table 3). In the enrichment capacity of Cu and Cd, Sedum plumbizincicola and Setaria lutescens showed the highest and lowest absorption capacity for Cu and Cd, respectively. The Cu and Cd concentrations in Sedum plumbizincicola were 451.5 mg·kg^−1^ and Cd 13.7 mg·kg^−1^, which were 13.8 and 11.8 times that in Setaria lutescens, respectively (Figure 3).

As an effective and widely used remediation measure of soil heavy metal contamination, phytoremediation is considered to be an effective method to reduce the total amount of soil heavy metals over time [54]. Thus, “removal efficiency” always be used to evaluate the remediation capability during the phytoremediation, which could be calculated using tissue concentration and biomass produced [55]. Therefore, the removal efficiency of different plants was not only related to the concentration of heavy metals in plants but also depends on the biomass of plants. After considering biomass and Cu and Cd concentrations, Pennisetum sp. showed the greatest Cu and Cd removal efficiency, with the three-year cumulative amounts of 8.67 × 103 g hm^−2^ and 121 g hm^−2^, respectively (Table 3). Although the concentrations of Cu and Cd in Elsholtzia splendens and Sedum plumbizincicola were quite different, they had similar removal efficiency of Cu and Cd after integrating the biomass. Because of the low biomass and Cu and Cd concentration in Setaria lutescens, the accumulation of Setaria lutescens for Cu and Cd was the lowest, which implied that this native plant species had poor removal efficiency during the phytoremediation aided by micron hydroxyapatite. According to our study results and the living habits of different plants, we suggest that the intercropping of Sedum plumbizincicola and Pennisetum sp. or Elsholtzia splendens can be an efficient way of phytoremediation aided by amendments. However, this assumption needs to be verified by further field experiments.

Based on this study, in the practice of phytoremediation aided by chemical materials, plant species with high biomass are recommended as remediation plants in some special areas, where the pollutants cannot be cut off. The rationality is that most of the hyperaccumulators behave low biomass production and are difficult to rapidly remove pollutants than plants with high biomass [56]. If the toxicity of heavy metals in soil is low in areas without foreign pollutant input, hyperaccumulator plants can certainly be used as the preferred plants to remove more trace metals. Otherwise, plants with easy cultivation, rapid growth, and large biomass may be suitable for phytoremediation aided by amendments such as the energy plants [57]. These energy plants with high biomass have the benefit for ecology and economy through providing a good habitat for soil animals, birds, snakes, etc., and even generating electricity through biomass combustion [58]. Therefore, we recommend the energy plants such as Pennisetum sp. can be used as the remediation plants for phytoremediation aided by soil amendments. In order to further improve the remediation efficiency, it can be intercropped with hyperaccumulators such as Sedum plumbizincicola.

### 3.4. Correlation between Metal Bioavailability and Environmental Factor

In order to obtain the influencing factors of bioavailability of Cu and Cd and plant accumulation of Cu and Cd, we analyzed the correlation between CaCl_2_-Cu, CaCl_2_-Cu, DGT-Cu, DGT-Cd, shoots Cu and Cd, and the environmental factors. The results of correlation analysis showed that the bioavailability of Cu and Cd was significantly negatively correlated with pH, SOC, T-P, A-P, and A-K (Table 4). This may be due to the addition of micron hydroxyapatite to the contaminated soil, which not only increases the content of soil total phosphorus and available phosphorus but also improves soil pH, and the increase of pH can reduce the bioavailability of Cu and Cd in the soil, thus reducing the Cu and Cd concentrations in plants [59]. Therefore, the bioavailability of Cu and Cd in the soil is mainly related to the addition of micron hydroxyapatite. After the contaminated soil is remediated by micron hydroxyapatite and planting different plants, the vegetation restoration leads to a large number of dead branches and leaves enter the soil every year, after microbial decomposition, more humus is formed, thus increasing soil organic matter [60]. Although the vegetation restoration cannot increase the absolute content of soil potassium, the growth of grass, rhizosphere microbial activities, and decomposition of organic residues will form a large number of organic acids, phenolic substances, and inorganic acids, which can accelerate the transformation of insoluble K into available K and increase the content of available K in soil [61]. Therefore, SOC and available K are significantly correlated with the bioavailability of Cu and Cd, but this correlation does not indicate that they can affect the bioavailability of Cu and Cd in soil. The biomass of plants was significantly negatively correlated with the bioavailability of Cu and Cd in soil but significant positive correlated with soil pH and SOC (Table 4). The addition of micron hydroxyapatite to the contaminated soil can reduce the bioavailability of Cu and Cd and increase the soil pH, which promote the growth of plants, thus promoting the accumulation of SOC. The accumulation of Cu and Cd is the result of the combined action of the soil bioavailability of Cu and Cd and biomass.

SOC, soil organic carbon; T-N, soil total nitrogen; A-N, available nitrogen; T-P, soil total phosphorus; A-P, available phosphorus; T-K, total potassium; A-K, available potassium; CEC, cation exchange capacity; T-Cu, total Cu; T-Cd, total Cd; C-Cu, CaCl_2_-extractable Cu; C-Cd, CaCl_2_-extractable Cd; D-Cu, DGT-extractable Cu; D-Cd, DGT-extractable Cd; P-Cu, Cu in plant; P-Cd, Cd in plant; A-Cu, plant Cu accumulation; and A-Cd, plant Cd accumulation. All samples of all plots included in these correlation analyses (*n* = 45). *P* < 0.05 correlation is significant at the 0.01 level; ^*∗*^ correlation is significant at the 0.05 level.

## 4. Conclusion

Results showed that the addition of micron hydroxyapatite promoted the growth of Setaria pumila, Pennisetum sp., Sedum plumbizincicola, and Elsholtzia splendens. At the same time, four plants combined with micron hydroxyapatite significantly increased soil pH, SOC, and decreased Cu and Cd fractions extracted by CaCl_2_ and diffusive gradients in thin films (DGT) than the untreated soils, respectively. Moreover, Pennisetum sp. has the maximum reduction for bioavailable Cu, Cd, and largest accumulation of Cu and Cd compared with other three plants. In general, the bioavailability of Cu and Cd in Pennisetum sp. treatment was the lowest than the other treatments. Thus, Pennisetum sp. (an energy plant) with high biomass is recommended as phytoremediation aided by soil amendments.

## Figures and Tables

**Figure 1:** Total Cu and Cd concentrations in five soils during 3 years. MW = Setaria lutescens, ME = Elsholtzia splendens, MS = Sedum plumbizincicola, and MP = Pennisetum sp. Different lowercase letters indicate significant differences in the same treatment during the three years (*n* = 3, *P* < 0.05).

**Figure 2:** CaCl_2_-extractable Cu and Cd and CDGT Cu and Cd in soils during 3 years. MW = Setaria lutescens, ME = Elsholtzia splendens, MS = Sedum plumbizincicola, and MP = Pennisetum sp. Different lowercase letters indicate significant differences in the same treatment during the three years (*n* = 3, *P* < 0.05).

**Figure 3:** Concentrations of (a) Cu and (b) Cd in the shoots of each plant. MW = Setaria lutescens, ME = Elsholtzia splendens, MS = Sedum plumbizincicola, MP = Pennisetum sp. Different lowercase letters indicate significant differences in the same treatment during the three years (*n* = 3, *P* < 0.05).

**Table 1:** Physicochemical properties of the tested soil.

pH	SOC g kg^−1^	T-N g kg^−1^	A-N mg kg^−1^	T-P g kg^−1^	A-P mg kg^−1^	T-K g kg^−1^	A-K mg kg^−1^	CEC cmol kg^−1^	T-Cu mg kg^−1^	T-Cd mg kg^−1^
4.24	16.5	1.08	54.0	0.190	89.4	2.02	51.1	8.31	666	0.412

SOC, soil organic carbon; T-N, soil total nitrogen; A-N, available nitrogen; T-P, soil total phosphorus; A-P, available phosphorus; T-K, total potassium; A-K, available potassium; CEC, cation exchange capacity; T-Cu, total Cu; and T-Cd, total Cd.

**Table 2:** Surface soil properties after the harvest of four plant species during the three years.

Time	Treatment	pH	SOC g kg^−1^	T-N g kg^−1^	A-N mg kg^−1^	T-P g kg^−1^	A-P mg kg^−1^	T-K g kg^−1^	A-K mg kg^−1^	CEC cmol kg^−1^
2013	CK	4.24 ± 0.207b	16.2 ± 0.191a	1.11 ± 0.0379a	52.5 ± 7.85a	0.190 ± 0.0100b	86.9 ± 1.71c	2.06 ± 0.140a	51.6 ± 2.98b	8.32 ± 0.0153a
	MW	5.17 ± 0.118a	16.3 ± 0.0458a	1.36 ± 0.0666a	54.8 ± 4.31a	0.620 ± 0.0872a	120 ± 7.26b	2.25 ± 0.0800a	94.3 ± 6.97a	8.41 ± 0.149a
	ME	5.33 ± 0.0503a	17.8 ± 0.398a	1.32 ± 0.0900a	55.8 ± 12.6a	0.650 ± 0.0306a	170 ± 9.12a	2.14 ± 0.164a	82.4 ± 15.1ab	8.63 ± 1.15a
	MS	5.19 ± 0.102a	18.0 ± 0.508a	1.26 ± 0.104a	52.6 ± 1.16a	0.780 ± 0.0723a	152 ± 5.89a	2.32 ± 0.0851a	94.7 ± 12.6a	7.84 ± 0.974a
	MP	5.15 ± 0.135a	18.0 ± 1.39a	1.27 ± 0.173a	52.5 ± 3.01a	0.710 ± 0.202a	149 ± 15.8a	2.07 ± 0.135a	71.7 ± 20.4ab	8.65 ± 0.575a

2014	CK	4.23 ± 0.110b	16.1 ± 0.172 b	1.05 ± 0.0306a	52.8 ± 7.06a	0.190 ± 0.0379b	88.1 ± 15.3b	1.97 ± 0.121b	49.5 ± 3.28b	8.39 ± 0.0404a
	MW	5.16 ± 0.130a	16.2 ± 0.118b	1.40 ± 0.0305a	56.3 ± 1.79a	0.620 ± 0.0764b	120 ± 10.2a	2.33 ± 0.0839a	98.0 ± 5.66a	8.53 ± 0.285a
	ME	5.24 ± 0.261a	18.4 ± 0.725a	1.33 ± 0.112a	56.4 ± 14.1a	0.520 ± 0.0404a	134 ± 3.60a	2.16 ± 0.159ab	84.0 ± 15.0ab	8.64 ± 0.710a
	MS	5.13 ± 0.195a	18.4 ± 0.239a	1.25 ± 0.123a	53.0 ± 0.197a	0.680 ± 0.0608a	132 ± 4.90a	2.31 ± 0.114ab	95.6 ± 13.4a	8.47 ± 0.180a
	MP	5.14 ± 0.253a	18.8 ± 0.546a	1.27 ± 0.251a	52.2 ± 2.47a	0.630 ± 0.242a	128 ± 3.27a	2.07 ± 0.147ab	72.0 ± 20.5ab	8.56 ± 0.206a

2015	CK	4.20 ± 0.280b	16.5 ± 0.451b	1.08 ± 0.0600b	54.0 ± 7.00a	0.190 ± 0.0153b	89.4 ± 4.02b	2.02 ± 0.0945c	51.1 ± 3.57b	8.36 ± 0.140b
	MW	5.03 ± 0.137a	16.6 ± 0.358b	1.45 ± 0.0379a	58.9 ± 3.70a	0.510 ± 0.136a	98.0 ± 5.70ab	2.43 ± 0.0265a	103 ± 5.12a	8.51 ± 0.0929b
	ME	5.26 ± 0.172a	19.0 ± 0.593a	1.46 ± 0.0436a	61.7 ± 11.9a	0.460 ± 0.0252ab	118 ± 5.16a	2.38 ± 0.0802ab	92.5 ± 12.9a	8.84 ± 0.071a
	MS	5.13 ± 0.161a	18.6 ± 1.09a	1.28 ± 0.0751ab	54.1 ± 2.05a	0.620 ± 0.102a	119 ± 11.5a	2.39 ± 0.0322ab	99.3 ± 16.8a	8.53 ± 0.0200b
	MP	5.07 ± 0.0971a	19.5 ± 0.478a	1.35 ± 0.276ab	55.5 ± 2.00a	0.550 ± 0.140a	116 ± 14.2a	2.20 ± 0.128bc	76.5 ± 19.1ab	8.56 ± 0.0819b

CK = untreated soil, MW = hydroxyapatite + Setaria lutescens, ME = hydroxyapatite + Elsholtzia splendens, MS = hydroxyapatite + Sedum plumbizincicola, MP = hydroxyapatite + Pennisetum sp. SOC, soil organic carbon; T-N, total nitrogen; T-P, total phosphorus; T-K, total potassium; A-N, available nitrogen; A-P, available phosphorus; A-K, available potassium; and CEC, cation exchange capacity. Different lowercase letters indicate significant differences between treatments at the same time (*n* = 3, *P* < 0.05).

**Table 3:** Shoot biomass and Cu and Cd accumulation in each plant during phytoextraction.

Treatment	Shoot biomass (t·hm^−2^)			Metal accumulation (g·hm^−2^)					
							Cu	Cd
	2013	2014	2015	2013	2014	2015	2013	2014	2015
CK	—	—	—	—	—	—	—	—	—
MW	10.1 ± 4.91bc	8.55 ± 1.52bc	5.20 ± 0.560c	236 ± 148c	285 ± 20.5b	224 ± 93.2b	10.4 ± 3.96b	10.3 ± 4.27b	6.50 ± 2.23c
ME	15.1 ± 4.17ab	12.6 ± 1.38b	14.4 ± 4.22b	2.74 × 103 ± 437a	2.54 × 103 ± 759a	2.93 × 103 ± 1.28 × 103a	39.2 ± 15.0a	32.1 ± 8.59a	37.6 ± 8.49b
MS	2.25 ± 0.365c	2.10 ± 0.210c	2.70 ± 0.468c	1.03 × 103 ± 266c	910 ± 92.8b	1.28 × 103 ± 395ab	29.8 ± 3.94ab	29.5 ± 1.10a	38.1 ± 5.15ab
MP	22.3 ± 3.36a	29.2 ± 6.10a	37.7 ± 4.14a	1.88 × 103 ± 353b	2.98 × 103 ± 949a	3.81 × 103 ± 1.40 × 103a	29.1 ± 4.46ab	39.8 ± 8.97a	52.0 ± 3.94a

CK = untreated soil, MW = hydroxyapatite + Setaria lutescens, ME = hydroxyapatite + Elsholtzia splendens, MS = hydroxyapatite + Sedum plumbizincicola, MP = hydroxyapatite + Pennisetum sp. Different lowercase letters indicate significant differences between treatments in the same year (*n* = 3, *P* < 0.05). — indicates no plant growth.

**Table 4:** Correlation coefficients among soil properties, Cu and Cd bioavailability, and remediation efficiency.

	pH	SOC	T-N	A-N	T-P	A-P	T-K	A-K	CEC	T-Cu	T-Cd	C-Cu	C-Cd	D-Cu	D-Cd	Biomass	P-Cu	P-Cd	A-Cu	A-Cd
PH	1.00																			
SOC	0.484^*∗∗*^	1.00																		
T-N	0.559^*∗∗*^	0.295^*∗*^	1.00																	
A-N	0.152	−0.0410	0.383^*∗∗*^	1.00																
T-P	0.699^*∗∗*^	0.396^*∗∗*^	0.580^*∗∗*^	−0.0430	1.00															
A-P	0.689^*∗∗*^	0.470^*∗∗*^	0.270	−0.121	0.691^*∗∗*^	1.00														
T-K	0.488^*∗∗*^	0.154	0.633^*∗∗*^	0.428^*∗∗*^	0.505^*∗∗*^	0.0690	1.00													
A-K	0.654^*∗∗*^	0.180	0.529^*∗∗*^	0.268	0.674^*∗∗*^	0.284	0.804^*∗∗*^	1.00												
CEC	0.225	0.162	0.0310	−0.0510	−0.146	0.110	−0.152	−0.106	1.00											
T-Cu	−0.538^*∗∗*^	−0.534^*∗∗*^	−0.225	−0.280	−0.330^*∗*^	−0.467^*∗∗*^	−0.374^*∗*^	−0.436^*∗∗*^	−0.0440	1.00										
T-Cd	−0.479^*∗∗*^	−0.609^*∗∗*^	−0.0520	−0.0810	−0.338^*∗*^	−0.220	−0.285	−0.397^*∗∗*^	−0.135	0.270	1.00									
C-Cu	−0.759^*∗∗*^	−0.414^*∗∗*^	−0.455^*∗∗*^	−0.0870	−0.798^*∗∗*^	−0.697^*∗∗*^	−0.444^*∗∗*^	−0.599^*∗∗*^	−0.0490	0.470^*∗∗*^	0.367^*∗*^	1.00								
C-Cd	−0.643^*∗∗*^	−0.355^*∗*^	−0.149	−0.0210	−0.673^*∗∗*^	−0.669^*∗∗*^	−0.217	−0.460^*∗∗*^	0.0660	0.356^*∗*^	0.480^*∗∗*^	0.826^*∗∗*^	1.00							
DGT-Cu	−0.813^*∗∗*^	−0.545^*∗∗*^	−0.580^*∗∗*^	0.0110	−0.789^*∗∗*^	−0.783^*∗∗*^	−0.303^*∗*^	−0.547^*∗∗*^	−0.0960	0.527^*∗∗*^	0.274	0.844^*∗∗*^	0.677^*∗∗*^	1.00						
DGT-Cd	−0.830^*∗∗*^	−0.509^*∗∗*^	−0.588^*∗∗*^	0.0420	−0.829^*∗∗*^	−0.723^*∗∗*^	−0.358^*∗*^	-0.624^*∗∗*^	−0.0350	0.404^*∗∗*^	0.345^*∗*^	0.794^*∗∗*^	0.733^*∗∗*^	0.938^*∗∗*^	1.00					
Biomass	0.44^*∗∗*^	0.548^*∗∗*^	0.243	−0.0150	0.321^*∗*^	0.335^*∗*^	−0.108	0.0450	0.301^*∗*^	−0.141	−0.454^*∗∗*^	−0.410^*∗∗*^	−0.358^*∗*^	−0.478^*∗∗*^	−0.498^*∗∗*^	1.00				
Plant Cu	0.438^*∗∗*^	0.563^*∗∗*^	0.122	−0.100	0.514^*∗∗*^	0.489^*∗∗*^	0.455^*∗∗*^	0.463^*∗∗*^	−0.169	−0.553^*∗∗*^	−0.472^*∗∗*^	−0.441^*∗∗*^	−0.472^*∗∗*^	−0.415^*∗∗*^	−0.408^*∗∗*^	−0.149	1.00			
Plant Cd	0.346^*∗*^	0.310^*∗*^	0.0230	−0.122	0.426^*∗∗*^	0.328^*∗*^	0.423^*∗∗*^	0.400^*∗∗*^	−0.0690	−0.295	−0.426^*∗∗*^	−0.340^*∗*^	−0.407^*∗∗*^	−0.244	−0.262	−0.268	0.852^*∗∗*^	1.00		
A-Cu	0.517^*∗∗*^	0.770^*∗∗*^	0.195	−0.0200	0.314^*∗*^	0.459^*∗∗*^	0.0400	0.148	0.241	−0.510^*∗∗*^	−0.580^*∗∗*^	−0.433^*∗∗*^	−0.404^*∗∗*^	−0.531^*∗∗*^	−0.503^*∗∗*^	0.790^*∗∗*^	0.295^*∗*^	0.0160	1.00	
A-Cd	0.595^*∗∗*^	0.738^*∗∗*^	0.216	−0.110	0.476^*∗∗*^	0.524^*∗∗*^	0.128	0.233	0.357^*∗*^	−0.406^*∗∗*^	−0.693^*∗∗*^	−0.502^*∗∗*^	−0.499^*∗∗*^	−0.527^*∗∗*^	−0.541^*∗∗*^	0.707^*∗∗*^	0.442^*∗∗*^	0.398^*∗∗*^	0.791^*∗∗*^	1.00

## Data Availability

All the data used to support the findings of this study are available from the corresponding author upon request.
